# The Impact of Digital Economy of Resource-Based City on Carbon Emissions Trading by Blockchain Technology

**DOI:** 10.1155/2022/6366061

**Published:** 2022-06-15

**Authors:** Jiahao Zhang, Jingyi Li, Duoduo Ye, Chuanqing Sun

**Affiliations:** ^1^School of Economics, Shanghai University, Shanghai City 200444, China; ^2^School of Management, Shanghai University, Shanghai City 200444, China; ^3^School of Management, Guangdong University of Technology, Guangzhou City 510006, China

## Abstract

To reduce the carbon emission intensity of resource-based cities and strengthen the sustainable development of these cities, firstly, blockchain technology is analyzed. Secondly, the development of the digital economy is discussed in digital resource-based cities. Finally, according to blockchain technology, a model of carbon emissions trading in the digital economy is designed, and the specific impact of the digital economy on carbon emissions trading is studied according to the model. The research results show that the mean value of the development index of the digital economy (*digital*) is −0.0168, the maximum value is 4.2560, the minimum value is −1.3429, and the standard deviation is 0.9572, indicating that the quality of digital economy development varies greatly among different regions. And according to the results of the digital model, it is found that the regression coefficient of the variable *digital* is significantly negative at the 1% level, showing that the digital economy will obviously suppress the carbon emission intensity of cities. After replacing the explained variables, the coefficient of the digital economy is still significantly negative. It indicates that the development of the digital economy can effectively suppress the carbon emission intensity of urban. Therefore, the designed model of carbon emissions trading under the blockchain technology can not only provide a secure platform for carbon emissions trading but also provide more comprehensive trading reference information for carbon emissions trading. It provides technical support for reducing the carbon emission intensity of resource-based cities and also contributes to the development of resource-based cities.

## 1. Introduction

Currently, under the premise of the rapid development of technology, blockchain, as an important channel for online transactions, provides users with an open, transparent, safe reliable, and traceable large-throughput platform at any time. The construction of blockchain technology provides a reliable platform for the development of the digital economy [1]. Nowadays, the development of resource-based cities urgently needs to solve the huge problem of carbon emissions trading. A resource-based city is a type of city in which the mining and processing of natural resources such as minerals and forests in the region are the leading industries. The cities are closely related to the production and development of cities and resource development. According to the sequence of resource exploitation and city formation, there are two modes for the formation of these cities. One is “mine first, then city”; that is, cities emerge entirely because of resource mining. The other is the “city first and then mine”; namely, the city existed before the resource development, and the resource development accelerated the city's development. The digital economy, supported by blockchain technology, provides good technical support for carbon emission trading in resource-based cities and also provides a reference for reducing the carbon emission intensity in resource-based cities [2]. Although carbon emissions trading has not been well solved at present, many studies have provided it with a technical reference.

Saberi et al. [3] pointed out that blockchain technology is on the ascendant in various fields as a technology of the distributed shared database. The decentralization, transparency, fairness, and openness of blockchain technology are in line with the concept of the energy Internet, and its application in the energy Internet will further promote the construction of the energy Internet. Litvinenko [4] proposed that in the context of economic globalization, the transformation of Information and Communications Technology (ICT) has been recognized as two important features of world economic development since the 1990s. The rapid development of ICT and the Internet has greatly accelerated the pace of economic globalization and promoted the increase in the scale and form of transnational trade in goods and services and international capital flows. The digital economy has become the mainstream of the world economy and the engine of economic growth. Sturgeon [5] indicated that the digital economy will become a new momentum for the development of China's economy under the new normal and an important force leading the national innovation strategy. China's development of the digital economy has the advantage of netizens, the late-mover advantage of achieving leapfrog development, and the institutional advantages of guaranteeing the organizational system. From the construction of high-speed ubiquitous information infrastructure and the digital economy to become an important engine of national economic development and fully integrate into production, China's digital economy is sailing and will certainly make greater contributions to global economic development. Chen and Lin [6] represented that the greenhouse effect is an important cause of global warming, and carbon dioxide is the most significant greenhouse gas in the greenhouse effect. Carbon emissions trading is a crucial measure to mitigate the greenhouse effect, and it is also one of the hotspots of current scientific research. Zhang et al. [7] expressed that the trading products of different carbon emission trading markets according to the types of greenhouse gas emission certificates can be divided into carbon emission allowances and carbon emission reductions certified. With the purpose of the carbon emissions trading market becoming more active and the continuous improvement of the trading mechanism, the interaction between the prices of different products has become increasingly close. How to recognize and utilize the relationship between product prices plays a vital role in grasping the price signals of the carbon market in a timely manner, reasonably selecting the types of trading products at different stages, and stabilizing and regulating the operation of the market. It can be found from the above research that the relevant research on carbon emissions trading is the main driving force for the sustainable development of resource-based cities in the future, but the current research in this area is not perfect, and there is no suitable trading platform for carbon emissions trading. Meanwhile, as a new type of science and technology with multiple advantages, blockchain can provide important technical support for carbon emissions trading.

To sum up, firstly, blockchain technology is discussed in depth, and secondly, the development prospects and functions of the digital economy are expounded. Finally, a model of the carbon emissions trading in the development of the digital economy is established based on blockchain technology, and the impact of the digital economy on carbon emissions trading is studied. The innovation lies in the use of new blockchain technology to provide innovative technical support for carbon emission trading in resource-based cities. This research provides a reference for the development of carbon emissions trading in resource-based cities and also contributes to the sustainable development of these cities.

## 2. Theory and Method

### 2.1. Blockchain Technology

A blockchain is a chain consisting of one block after another. Each block stores a certain amount of information, and they are connected into a chain according to the time sequence of their generation. This chain is kept in all servers, and as long as one server in the entire system can work, the entire blockchain is secure. These servers are called nodes in the blockchain system, and they provide storage space and computing power support for the entire blockchain system.

Blockchain is a distributed general ledger system. Transactions in the blockchain system are open, transparent, and traceable. They are usually used in encrypted file transmission and economic transactions. During the transaction process, both parties to the transaction can trade anonymously and encrypt files, so its main characteristics are security and timing. Blockchain technology is actually a database that can store data distributedly and establish more advanced computer technologies such as smart contracts, encryption algorithms, and consensus mechanisms [8]. On the whole, blockchain technology means that everyone participates in the transaction process. When a transaction is carried out, everyone can witness and record, and the system will also record transactions and store them in partitions. When all transactions are recorded and stored in partitions and then connected together with everyone, the backup is collectively referred to as the blockchain [9].

Blockchain has the characteristics of decentralization, trustless, encryption security, and traceability. Among them, decentralization means that the system is built by the central node, which controls and publishes management decisions. However, the essence of blockchain is a distributed consensus system; that is, transactions between users do not need the agents of the central node but directly trade and interact between users [10]. Decentralization makes the trading model of transaction blockchain larger and more efficient and information transmission faster and removes intermediary agency mechanisms to help transactions easier [11].

The trustless characteristic does not mean that the blockchain system does not need trust, but that blockchain makes the transaction trust mechanism more secure in the blockchain system through rules, technologies, and algorithms [12]. Blockchain technology is different from traditional Internet technology. Transactions in blockchain systems do not need to understand the information of the counterparty, to determine its trust limit. Instead, it relies on the algorithm of blockchain to establish an anonymous trading system, which can fully protect the reasonable and legitimate rights and interests of the trader, thus promoting the secure transaction process of blockchain [13].

The feature of encryption security means that the transaction process under the blockchain system needs to be authenticated. The blockchain uses the hash value to match the blocks in the transaction process. If the transaction content changes during the transaction process, the hash value cannot match, and the transaction content will lose its meaning [14]. The blockchain is to record the practice signature on the blockchain and then use the time stamp to record and check the transaction content of both parties. If the accounting content does not match, the blockchain will prevent the transaction from proceeding, thereby reducing the occurrence of illegal acts such as fraud [15].

The feature of traceability means that every transaction conducted in the blockchain will be recorded in the blockchain system, the details of each transaction will be recorded, and the link will be sorted according to the time the transaction occurred, forming a blockchain by combining the information link of each transaction. In the blockchain, this data information will be stored in a block structure with time tags. Each transaction can be traced and verified, which is quite efficient in verifying the use of funds and information leakage [16]. The basic principle and system framework of blockchain technology are shown in Figure 1.

In Figure 1, trading in the blockchain is peer-to-peer interaction, and it is transparent, open, secure, and traceable enough. Currently, blockchain technology is divided into three types. One is the public type; that is, there is no network center node in the blockchain trading system at all, but a transparent and open peer-to-peer trading system [17]. The second is the private type; that is, blockchain technology is controlled and managed by developers. Transactions in the system will be managed and audited by developers, and public modes can be set up, to set up an internal trust system [18]. The third is the alliance type, which means that a consensus is reached in the form of an alliance, and the alliance mechanism of multiple systems is formed with the authorization of the developers and is jointly managed and controlled by multiple nodes to jointly promote the operation of the blockchain [19]. Due to the outstanding transaction advantages of blockchain, it has been called the main transaction method in current economic transactions [20].

### 2.2. Digital Economy of Resource-Based City

Resource-based cities refer to cities with sustainable development and resources used by human beings [21]. Resources refer to the general term for all material, information, and energy that can be discovered and used by human beings. Resources exist anywhere and can be used to create wealth and value for human beings [22]. The narrow interpretation of resources means natural resources, but not all-natural substances surrounding human beings are natural resources, but substances in nature that can create economic value for human beings under certain time and place conditions. Natural resources are classified into depleted, renewable, and sustainable natural resources. The sustainable consumption of natural resources refers to the regeneration rate being very fast, can be regenerated within a certain period of time, and has little or no impact on the subsequent consumption and use of human beings [23]. Renewable resources refer to natural resources that are regenerated quickly and can self-recover within a certain period of time. If developed and used later, it will have a certain impact on their recovery activities [24]. Depleted resources refer to the relatively slow regeneration rate and need to be generated through long-term geological accumulation, so there will be depletion in the process of human use, that is, natural resources that continue to be used with human use and have only one chance of use in human history [25]. The broad meaning of resources includes not only the resources of nature but also the human resources in human society. Social and human resources are the general term for resources composed of social wealth and material wealth generated by human beings engaged in social and economic activities [26]. The principles of narrow and broad resources are shown in Figure 2.

In Figure 2, broad and narrow resources together constitute all the resources that can be used and bring wealth to mankind in human society. Resource-based cities economy refers to the use of resources in the city to form an economic growth model with resource exploration and primary processing as important industries. Resource-based cities' economy mainly relies on the exploration and utilization of depleted resources and the formation of industrial clusters on a secondary basis. Under this economic model, resources replace the main force of production in other industries such as capital, labor, and technology [27]. However, with the consumption of resources, when the resources are not recovered or the recovery is too slow and the supply is insufficient, this economic industrial chain will break, this resource-based economic model will also go bankrupt, and resource-based cities will also face the scene of economic scarcity with the depletion of resources. Meanwhile, in the process of resource development, it will not only cause certain damage to the urban environment but also cause an irreversible negative impact on the daily life of citizens. Therefore, the resource-based cities economy will go through the process of “the rise of resource-based industries-the dominance of resource-based industries - the decline of resource-based industries - the decline or transformation of resource-based cities”. The digital economy is a virtual economic model produced by Internet technology as the main technology. Because the Internet has efficient computing speed and large-scale transmission capacity, it can provide major technical support for the development of the digital economy. To a certain extent, the digital economy is the phenomenon of economic networking and globalization through digital technologies such as the Internet, so the digital economy has become the main trend in contemporary cities' economic development [28].

### 2.3. Carbon Emissions Trading

Carbon emission trading refers to the determination of the right to discharge pollutants and the total amount of emissions within a certain period of time within an area under the effective jurisdiction of the government. The emission rights can be traded in the market as permitted by law. In this way, carbon emission rights can be traded with ordinary commodities in the market, and the total amount of pollutants can be coordinated. Finally, the lowest-cost emission reduction target can be achieved within the total emission limit that does not exceed the legal limit [29]. The main purpose of carbon emission trading is to solve environmental problems, especially the negative impact of climate change caused by emissions, but this negative impact is not reflected in transaction costs and transaction prices. The basic principle of carbon emission rights trading has good practicality. Compared with the general carbon emission mechanism, the trading method of carbon emission rights can not only reduce the cost of pollution discharge but also improve the efficiency of pollution discharge. Currently, the carbon emission trading system includes two methods, the baseline emission reduction and credit trading system and the total control and trading system [30]. Among them, the total control and trading system refers to the total amount of emissions by setting a limited and tradable emission quota, and in the process of emission, it is necessary to ensure that the amount of emission of each emission system cannot exceed its quota. Under this system, enterprises will choose to reduce the number of pollutants discharged by the enterprise to reduce the cost of pollutant discharge from the full use of quotas and reduction of emissions. But when the carbon emission allowance is sufficient and the emission cost is fixed, the enterprise will make full use of the emission allowance to realize its maximum value, so the limited allowance will make the enterprise reduce the emission and save its own economy. In this system, government agencies that manage the emission process need to allocate emission quotas reasonably and allow emission rights to be traded, to ensure emission reductions and save emission costs. The baseline emission reduction and credit trading system refers to emission reduction actions generated through emission reduction projects. The carbon emission trading system needs to be connected; that is, one carbon emission system uses the units of another emission system to achieve the main purpose of carbon emission. Its main purpose is to reduce the cost of carbon emission reduction, increase market liquidity, and support cooperation on climate change. The cooperation of emission trading rights will not only bring benefits to both parties but also play an exemplary role for other cities [31]. The specific principle of carbon emission trading is shown in Figure 3.

In Figure 3, under the quota allocation of the city manager, the enterprise obtains the emission quota and obtains the right to trade it, and then the enterprise has the right to discharge its own pollutants, which reflects the value of the quota. Meanwhile, they can also trade quotas, obtain the benefits brought by quotas, and transfer pollutant discharge rights, so that enterprises that need the power to discharge pollutants can obtain sufficient quotas to complete the process of discharging pollutants.

## 3. Digital Economy and Carbon Emission Trading Model by Blockchain

### 3.1. The Trading Model of Digital Economy of Blockchain

The features of openness, transparency, encryption security, and traceability of blockchain technology can provide an important guarantee for the transaction process of the digital economy. Therefore, it is a very important choice to use blockchain technology to trade in the process of carbon emission trading. Through blockchain technology, quotas of enterprise emissions are publicly released by government agencies, and then enterprises can use them or find other enterprises in the blockchain system to trade. Blockchain technology can provide buyers with transparent information not only to help them obtain transaction information but also to ensure that buyers will not be cheated during the transaction process. For sellers, they can trade openly, obtain transparent trading value, and ensure their legal and safe access to benefits through the trading method of the digital economy. Therefore, blockchain technology not only improves the safety of the carbon emission trading process but also provides a significant reference platform to be reasonably used for carbon emission quotas. The model principle of digital economy trading and carbon emission trading through blockchain technology is shown in Figure 4.

In Figure 4, the open and transparent feature of blockchain provides favorable information for both parties to the transaction. The feature of encrypted security provides transaction protection for the transaction process of both parties, helping both parties to trade smoothly and maximizing the interests of both parties. Traceability can help all participants to find all information, and timely traceability can provide the final transaction guarantee for both parties to the transaction and government agencies. Through blockchain technology, the impact of the digital economy of resource-based cities is studied on carbon emission trading in the digital economy and carbon emission trading, to standardize carbon emissions of cities, protect the cities' environment, slow down the resource utilization process of resource-based cities, and promote the long-term development of resource-based cities.

### 3.2. Model of the Impact of the Digital Economy on Carbon Emission Trading

The natural logarithm of carbon emission intensity is selected as the interpreted variable to measure the carbon emission level of cities. The carbon emission intensity is obtained by calculating the carbon emissions of cities divided by the real GDP of the region in the current year (the nominal GDP of the region is equalized in 2011 as the base period) [32]. The calculation is shown in

(1) $$\begin{array}{c} intensity_{i,t}=\frac{emission_{i,t}}{G\;DP_{i,t}}. \end{array}$$

In (1), **intensity**_*i*,*t*_ indicates the carbon emission intensity of the **t** th year of the **i** th city. **emission**_*i*,*t*_ shows the carbon emissions, and **G**  **DP**_**i**,**t**_ means the real GDP of the **t** th year of the **i** th city. Based on the impact of the digital economy on carbon emissions trading, a regression model and a mediating effect test model are built through the impact of the digital economy on the carbon emissions intensity of cities. The digital economy can curb the carbon emissions intensity of cities by promoting technological innovation and advanced industrial structure [33]. The model is shown in equations (2), (3), and (4):

(2) $$\begin{array}{c} lnintensity_{i,t}=\alpha_{0}+\alpha_{1}digital_{i,t}+\alpha_{2}control_{i,t}+city_{i}+year_{t}+\varepsilon_{i,t}, \end{array}$$

(3) $$\begin{array}{c} mediator_{i,t}=\beta_{0}+\beta_{1}digital_{i,t}+\beta_{2}control_{i,t}+city_{i}+year_{t}+\varepsilon_{i,t}, \end{array}$$

(4) $$\begin{array}{c} lnintensity_{i,t}=\theta_{0}+\theta_{1}digital_{i,t}+\theta_{2}me\;diator_{i,t}+\theta_{3}control_{i,t}+city_{i}+year_{t}+\varepsilon_{i,t}, \end{array}$$

where **i** is the city and **t** is the year. The explained variable **lnintensity**_*i*,*t*_ represents the carbon emission intensity, and the core explanatory variable **di**  **gital**_*i*,*t*_ represents the development level of the digital economy. **control**_**i**,**t**_ shows the control variable. **city**_*i*_ is the fixed effect of cities. **year**_*t*_ is the fixed effect of the time. *ε*_**i**,**t**_ is a random disturbance term. **me**  **di**  **ator**_*i*,*t*_ is a mediating variable, namely, technological innovation (**lnpatent**_*i*,*t*_) or industrial structure advanced ((**lnhigh**_*i*,*t*_)). Equation (2) is the total effect of the digital economy on the carbon emission intensity of cities, and its coefficient *α*_1_ represents the size of the total effect. In (3), the coefficient *β*_1_ indicates the influence of the digital economy on the mediating variable. In (4), the coefficient *θ*_1_ indicates the direct effect of the digital economy on carbon emission intensity, and the product *β*_1_*θ*_2 _ of the coefficient *θ*_2 _ and the coefficient *β*_1 _ in (3) means the size of the mediating effect; that is, the digital economy promotes technological innovation or the advanced industrial structure can reduce the influence coefficient of carbon emission intensity. If the regression coefficient *θ*_2 _ is significantly negative, it indicates that the carbon emission intensity of cities can be reduced by promoting technological innovation or the advanced industrial structure. If the absolute value of the regression coefficient *θ*_1 _ is both smaller than the absolute value of *α*_1_, it means that the two can play a mediating role in the process of suppressing carbon emission intensity in the digital economy. If *β*_1_*θ*_2_ and *θ*_1 _ have the same value, it means that the effect is a partial mediating effect [34].

### 3.3. Settings of Research Data

The designed model under the blockchain technology uses carbon emission trading data for evaluation. The main source of data is the Global Carbon Budget (GCB) database. The scientific goal of the GCB is to fully understand the global carbon cycle, including its characteristics and interactions, synthesize current understanding of the global carbon cycle, and provide rapid feedback to research institutions, governments, and the public. Regional/national carbon plans are provided a global coordination platform to enhance research on broader national and regional carbon research plans and projects in more related disciplines through better coordination, clear goals, and the development of conceptual frameworks. Databases detail all datasets and model results for carbon budgets, one for GCB and one for national-level emissions inventories. The carbon emission data in 2019 in the database and the budget data for future carbon emissions in the database are mainly used.

## 4. Carbon Emission Trading of Digital Economy in Resource-Based City

### 4.1. Relevant Research on Carbon Emission Trading of Resource-Based Cities

Through the research on the relevant data of carbon emission trading of the current resource-based cities, the development of carbon emission trading of the resource-based cities can be analyzed, and the prospect and development direction of carbon emissions trading can be analyzed specifically. The development status of resource-based cities is shown in Figure 5.

In Figure 5, *mean* represents the average value, *sd* refers to the sample standard deviation, max shows the maximum value, and min indicates the minimum value. The mean of the development index of the digital economy (*digital*) is −0.0168, the maximum value is 4.2560, the minimum value is −1.3429, and the standard deviation is 0.9572, indicating that the quality of digital economy development varies greatly among different regions. From the perspective of control variables, different prefecture-level cities also have obvious differences in terms of population density (people), urbanization level (urban), financial development level (fin), and invention patent authorization (patent). Therefore, to promote the sustainable development of resource-based cities, reasonable carbon emissions are necessary.

### 4.2. Carbon Emission Trading in the Digital Economy

As mentioned above, the reasonable disposal of carbon emissions is a necessary measure for the sustainable development of resource-based cities at present. Therefore, the trading of enterprise carbon emissions is studied according to the development foundation of the digital economy. With the support of blockchain technology, the transaction of carbon emission trading is more open, transparent, safe, and reliable, and the transaction can be traced at any time to prevent transaction chaos. The results of the benchmark regression of carbon emission intensity of the digital economy are shown in Table 1.

Column (2) shows the regression results obtained without considering control variables, and column (3) shows the regression results obtained after adding control variables. Each regression takes into account fixed effects of city and time and initially controls the endogenous problems caused by omitted variables. According to the regression results reported in Table 1, there is a significant negative correlation between the digital economy and carbon emission intensity at 1%, indicating that the development of the digital economy can significantly suppress carbon emission intensity. In addition, the scale of government spending (gov) is obviously positively correlated with carbon emission intensity at 1%, showing that reducing the scale of government spending can effectively reduce carbon emission intensity. Besides, it is necessary to examine the impact of the development of the digital economy on the carbon emission intensity of cities, to study the specific impact of the development of the digital economy on carbon emission sources. The results of the impact of digital economy development on the carbon emission intensity of cities are shown in Table 2.

In Table 2, it is obvious from the results in column (2) that the digital economy can significantly reduce the carbon emission intensity of cities. As shown in columns (3) and (4), it is not difficult to find that the influence coefficients of the digital economy on regional technological innovation and advanced industrial structure are significantly positive at the 1% level. This may be because, on the one hand, the development of the digital economy has reduced the financing debt problems of small and medium enterprises (SMEs) in the R&D process, thereby promoting the overall improvement of the regional technology level and realizing technological innovation. On the other hand, the digital economy has increased the proportion of clean industries and services, and the relative proportion of heavy industry has decreased. As a result, the industrial structure continues to develop to a higher stage. Columns (1) to (6) show that the estimated coefficients of *α*_1, *β*_1, and *θ*_2 of the model (2) to (4) above have all passed the significant test of 1%. It indicates that there are two ways for the digital economy to suppress the carbon emission intensity of cities: one is by promoting regional technological innovation, and the other is by promoting the upgrading of industrial structures. The Internet penetration rate and the interchange term between each city and Hangzhou are used as instrumental variables (IV) for further analysis. This IV meets the two basic conditions of correlation and exogenous: first, the Internet penetration rate represents the degree of digitalization in a region and has a strong correlation with the digital economy. The “distance between the city and Hangzhou” is directly related to the digital inclusive financial index (DIFI) of prefecture-level cities and then related to the digital economy. Second, neither the Internet penetration rate nor the “distance between the city and Hangzhou” can affect the carbon emission intensity and meet the exogenous conditions by affecting the digital economy. The regression results of the two stages are shown in Table 3.

The first-stage regression verifies the correlation between instrumental variables and the digital economy. The regression results in column (2) of Table 3 show that instrumental variables and endogenous explanatory variables are significantly correlated. Column (3) of Table 3 is the regression results of the second stage, which shows that the regression coefficient of the variable digital is significantly negative at the 1% level, indicating that the digital economy will significantly suppress the carbon emissions intensity of cities. The natural logarithm of carbon emission intensity (lnintensity) of the explained variable is replaced by the natural logarithm of carbon emission (lnemission), and the fixed effects of city and time are considered simultaneously. Following the constructed instrumental variables, the regression results are shown in column (4) of Table 3. After replacing the explained variables, the coefficient of the digital economy is still significantly negative. It means that the development of the digital economy can effectively suppress the carbon emissions intensity of cities.

## 5. Discussion

From the above results, it manifests that the average value of the development index of the digital economy (*digital*) is −0.0168, the maximum value is 4.2560, the minimum value is −1.3429, and the standard deviation is 0.9572, illustrating that the quality of digital economy development varies greatly among different regions. In addition, the maximum population density (People) of different prefecture-level cities is around 1500 people/km^2^, the minimum is around 90 people/km^2^, and the standard deviation is around 400 people/km^2^; the maximum urbanization level (Urban) is around 9. The minimum is around 4; the maximum of the financial development level (Fin) is around 3.2, and the minimum is around 0.3; the maximum of invention patent authorization (Patent) is around 6,000, and the minimum is around 5,000. It demonstrates that there are also obvious differences between different cities in terms of population density, urbanization level, financial development level, and invention patent authorization. Therefore, it can be seen that research on carbon emissions trading and balancing the development status of different cities will have a vital influence on the common development of cities in the future. According to the data analysis results in the GCB database, the digital economy is obviously negatively correlated with carbon emission intensity at the 1% level, which indicates that the development of the digital economy can significantly suppress carbon emission intensity. Furthermore, the scale of government spending (gov) is significantly positively correlated with carbon emission intensity at the 1% level, showing that reducing the scale of government spending can effectively reduce carbon emission intensity. It can be known that the digital has a vital effect on the development of carbon emissions trading. It is of great significance to study the development of urban carbon emissions trading through the digital economy. Meanwhile, the digital economy can provide important support for carbon emissions trading in the future. The influence coefficients of the digital economy on regional technological innovation and industrial structure upgrading are both remarkable positive at the 1% level. This may be because, on the one hand, its development has reduced the financing debt problems of small and medium-sized enterprises (SMEs) in the process of research and development, thereby promoting the overall improvement of the regional technology level and realizing technological innovation. On the other hand, it has increased the proportion of clean industries and service industries, while the relative proportion of heavy industry has decreased, thus making the industrial structure continue to develop to a higher level. Based on the above research results, firstly, it refers that the designed carbon emission trading model under the blockchain technology has multiple advantages, which can greatly guarantee the growth of the carbon emission trading industry. Secondly, driven by the digital economy, the carbon emission trading industry will develop more rapidly.

## 6. Conclusion

With the progress of society, carbon emissions have become the main driving force for the sustainable development of resource-based cities. Therefore, research and development of industries that promote carbon emissions trading play a critical role in society. Based on this, the impact of the development of the digital economy on the carbon emission trading of resource-based cities is studied under blockchain technology. The development of the digital economy has many advantages such as openness, transparency, safety, reliability, and traceability. Through the development of the digital economy, the carbon emission intensity of resource-based cities is analyzed, which has a strong impetus for the sustainable development of resource-based cities. The research shows that the current development trend of the digital economy is significantly different in each city, so driven by the current technological development, it is necessary for each resource-based city to focus on the development of the digital economy, and to discover the impact of the digital economy on resource-based cities. First, the digital economy can effectively reduce carbon emission intensity. Second, the digital economy can reduce carbon emission intensity by promoting regional technological innovation and advanced industrial structure. Third, compared with nonresource-based cities, the inhibitory effect of the digital economy on the carbon emission intensity of cities is more significant in resource-based cities. Further analysis shows that this inhibitory effect is more obvious in mature and declining resource-based cities. Although it provides sufficient data to prove the impact of the digital economy on carbon emissions trading, there is still a lack of research on practical applications. In the future, the practical application research on the impact of the digital economy on carbon emission trading will be strengthened.

## Figures and Tables

**Figure 1:** The basic principle and system framework of blockchain technology: (a) the structure of blockchain; (b) the transaction principle of blockchain.

**Figure 2:** Types of resources: (a) the narrow resource; (b) the broad resources.

**Figure 3:** Principles of carbon emissions trading.

**Figure 4:** Carbon emission trading of blockchain technology.

**Figure 5:** Development status of resource-based cities: (a) industry status; (b) economic status.

**Table 1:** The results of the benchmark regression of carbon emission intensity of the digital economy.

	(1)	(2)
	Lnintensity	Lnintensity
*Digital*	−0.2156 ^*∗*^ ^*∗*^ ^*∗*^	−0.1659 ^*∗*^ ^*∗*^ ^*∗*^
	(0.0056)	(0.0067)

*fdi*		2.9017
		(2.2716)

*People*		0.0002
		(0.0001)

*Urban*		−0.2796 ^*∗*^ ^*∗*^ ^*∗*^
		(0.0567)
*fin*		−0.0363 ^*∗*^ ^*∗*^
		(0.0171)

*gov*		0.3072 ^*∗*^ ^*∗*^ ^*∗*^
		(0.1155)

*intl*		−0.0267
		(0.0349)

*inv*		−0.4119 ^*∗*^ ^*∗*^ ^*∗*^
		(0.0216)

Constant	−13.3607 ^*∗*^ ^*∗*^ ^*∗*^	−11.5277 ^*∗*^ ^*∗*^ ^*∗*^
	(0.0261)	(0.2778)

City Fe	Yes	Yes
Year Fe	Yes	Yes
Adjusted *R*^2^	0.5068	0.6430
N	1680	1680

*Note.* ^*∗*^ ^*∗*^ ^*∗*^,  ^*∗*^ ^*∗*^, and  ^*∗*^ represent significant levels of 1%, 5%, and 10%, respectively, with robust standard errors in parentheses.

**Table 2:** The results of the impact of digital economy development on the carbon emission intensity of cities.

	(1)	(2)	(3)	(4)	(5)
	*Lnintensity*	*Lnpatent*	*Lnintensity*	*Lnhigh*	*Lnintensity*
*Digital*	−0.1659 ^*∗*^ ^*∗*^ ^*∗*^	0.5645 ^*∗*^ ^*∗*^ ^*∗*^	−0.1149 ^*∗*^ ^*∗*^ ^*∗*^	0.1381 ^*∗*^ ^*∗*^ ^*∗*^	−0.1544 ^*∗*^ ^*∗*^ ^*∗*^
	(0.0067)	(0.0275)	(0.0068)	(0.0087)	(0.0071)

*Lnpatent*			−0.0979 ^*∗*^ ^*∗*^ ^*∗*^		
			(0.0056)		

*Lnhigh*					−0.1038 ^*∗*^ ^*∗*^ ^*∗*^
					(0.0221)

Controls	Yes	Yes	Yes	Yes	Yes
Constant	−11.5277 ^*∗*^ ^*∗*^ ^*∗*^	−2.3221 ^*∗*^ ^*∗*^ ^*∗*^	−11.8239 ^*∗*^ ^*∗*^ ^*∗*^	−0.7174 ^*∗*^ ^*∗*^ ^*∗*^	−11.4392 ^*∗*^ ^*∗*^ ^*∗*^
	(0.2778)	(0.7603)	(0.2676)	(0.2441)	(0.2779)

City Fe	Yes	Yes	Yes	Yes	Yes
Year Fe	Yes	Yes	Yes	Yes	Yes
Adjusted *R*^2^	0.6430	0.4914	0.7075	0.4949	0.6487
N	1680	1680	1680	1680	1680

**Table 3:** The regression results of the two stages.

	First stage	Second stage	
	(1) digital	(2) lnintensity	(3) lnemission
IV	0.0041 ^*∗*^ ^*∗*^ ^*∗*^		
	(0.0002)		

Digital		−0.2989 ^*∗*^ ^*∗*^ ^*∗*^	−0.0102 ^*∗*^ ^*∗*^ ^*∗*^
		(0.0171)	(0.0036)

Controls	Yes	Yes	Yes
Constant	−6.1629 ^*∗*^ ^*∗*^	−11.0091 ^*∗*^ ^*∗*^ ^*∗*^	2.2823 ^*∗*^ ^*∗*^ ^*∗*^
	(2.7887)	(0.9249)	(0.2924)

City Fe	Yes	Yes	Yes
Year Fe	Yes	Yes	Yes
Adjusted *R*^2^	0.6116	0.5323	0.1357
N	1680	1680	1680

## Data Availability

The data used to support the findings of this study are included within the article.
